The article "Treatment of Coronal Plane Femoral Intertrochanteric Fractures with a Microexternal Fixator Combined with Proximal Femoral Nail Antirotation" was retracted in 2023. Reasons: signs of a paper mill; suspected computer-generated content; unreliable results or conclusions; concerns about the data.

# Treatment of Coronal Plane Femoral Intertrochanteric Fractures with a Microexternal Fixator Combined with Proximal Femoral Nail Antirotation

**DOI:** 10.1155/2022/1735603

**Published:** 2022-01-17

**Authors:** Mingke Zhou, Yuan Chen, Jun Qian, Yunji Zeng, Liangshan Huang, Yuanlei Zheng

**Affiliations:** ^1^Department of Orthopedics, Cangnan County Hospital of Traditional Chinese Medicine, Cangnan 325800, Zhejiang Province, China; ^2^Department of Orthopedics, Xinchang County Hospital of Traditional Chinese Medicine, Xinchang 312599, Zhejiang Province, China; ^3^Department of Orthopedics, Jinhua Fifth People's Hospital, Zhejiang Province 321399, China; ^4^Department of Orthopedics, The Affiliated Hospital of Hangzhou Normal University, Hangzhou 310015, Zhejiang Province, China

## Abstract

**Objective:**

To investigate the different efficacy of proximal femoral nail antirotation (PFNA) combined with or without a microexternal fixator in the treatment of coral-plane femoral intertrochanteric fractures.

**Methods:**

120 patients with intertrochanteric coronal fractures who received treatment in four hospitals from February 2020 to February 2021 were retrospectively included in this study. They were divided into control (PFNA alone, *n* = 60) and combined treatment group (a microexternal fixator + PFNA, *n* = 60) according to different surgery methods. All patients were followed up for 6 months. Operative time, amount of intraoperative blood loss, postoperative length of hospital stays, fracture healing time, Harris hip score, modified Barthel index, hip function excellent and good rate, and incidence of complications were compared between the two groups.

**Results:**

There were no significant differences in operative time, amount of intraoperative blood loss, postoperative length of hospital stay, and incidence of complications between the two groups (all *P* > 0.05). Fracture healing time in the combined treatment group was significantly shorter than that in the control group (*P* < 0.05). After surgery, Harris hip score and modified Barthel index in each group were significantly increased compared with before surgery (both *P* < 0.05). The increases in Harris hip score and modified Barthel index in the combined treatment group were significantly greater than those in the control group (both *P* < 0.05). After surgery, Harris hip function excellent and good rate in the combined treatment group was significantly higher than that in the control group (83.33% > 66.67%, *P* < 0.05).

**Conclusion:**

Compared with PFNA alone, a microexternal fixator combined with PFNA for the treatment of coronal plane femoral intertrochanteric fractures can greatly shorten fracture healing time and improve postoperative hip function and activities of living ability, but it cannot greatly increase operative time, the amount of intraoperative blood loss, or the risk of postoperative complications.

The article "Treatment of Coronal Plane Femoral Intertrochanteric Fractures with a Microexternal Fixator Combined with Proximal Femoral Nail Antirotation" was retracted in 2023. Reasons: signs of a paper mill; suspected computer-generated content; unreliable results or conclusions; concerns about the data.

## 1. Introduction

With the rapid increase of the aging population in China, femoral intertrochanteric fractures are a common type of clinical fractures, accounting for about 57.4% of hip fractures; coronal plane femoral intertrochanteric fractures are the main fracture type, accounting for approximately 88.4% [1–3]. They are extremely unstable and have difficulties in surgical fixation. Proximal femoral nail antirotation (PFNA) internal fixation is often used to manage coronal plane femoral intertrochanteric fractures, but internal fixation failure occurs in some patients, affecting prognosis [4, 5]. Therefore, it is of great significance to find a novel fracture reduction method and/or internal fixation instrument to reduce the incidence of internal fixation failure. Taking the data regarding clinical treatment of femoral intertrochanteric fractures collected by our team over many years as evidence, we designed a novel microexternal fixator composed of threaded Steinman's pins and a self-designed external fixation system after summarizing the literatures regarding coronal plane femoral intertrochanteric fractures. We treated coronal plane femoral intertrochanteric fractures with the self-designed microexternal fixator and investigated its preliminary therapeutic effects.

## 2. Materials and Methods

### 2.1. General Data

A total of 120 patients with coronal plane femoral intertrochanteric fractures who received treatment in Cangnan County Hospital of Traditional Chinese Medicine, Xinchang County Hospital of Traditional Chinese Medicine, Jinhua Fifth People's Hospital, and The Affiliated Hospital of Hangzhou Normal University, from February 2020 to February 2021, were included in this study. They were divided into control and combined treatment groups (*n* = 60/group) according to different surgery methods. In the control group, male-to-female ratio was 12 : 18, and the average age was (70.81 + 10.38) years. Causes of fracture included falls (*n* = 54) and traffic accidents (*n* = 6). Complications included diabetes mellitus (*n* = 4), hypertension (*n* = 9), and coronary heart disease (*n* = 6). In the combined treatment group, male-to-female ratio was 10 : 20, and the average age was (68.13 ± 11.34) years. Causes of fracture included falls (*n* = 52) and traffic accidents (*n* = 8). Complications included diabetes mellitus (*n* = 5), hypertension (*n* = 8), and coronary heart disease (*n* = 9). There were no significant differences in baseline data between the two groups. This study was approved by institutional ethics committee, and patients and their family members signed informed consent.

The article "Treatment of Coronal Plane Femoral Intertrochanteric Fractures with a Microexternal Fixator Combined with Proximal Femoral Nail Antirotation" was retracted in 2023. Reasons: signs of a paper mill; suspected computer-generated content; unreliable results or conclusions; concerns about the data.

### 2.2. Inclusion and Exclusion Criteria

The inclusion criteria are as follows: patients with coronal plane femoral intertrochanteric fractures confirmed by multiprojection CT scans [6], aged 60 years and older, indication of femoral intertrochanteric fractures on CT scans and AO/OTA type 31A2.2-31A2.3, fresh (within 2 weeks) fractures, and those who have good health and were able to tolerate surgery and anesthesia. The exclusion criteria are as follows: patients with femoral intertrochanteric fractures not involving coronal plane fractures, pathological fracture, open fracture, those having a previous history of hip surgery or abnormal hip function, and those with severe heart, liver, kidney diseases, or infectious diseases.

### 2.3. Methods

In both groups, patients underwent preoperative preparation. For patients who had complications, their blood pressure, blood glucose, and heart rate were controlled to be within the normal range. In the control group, patients received PFNA internal fixation. Precisely, patients were taken to lie on the orthopedic traction bed. After general anesthesia, closed reduction was conducted under a mobile C-arm X-ray fluoroscopy machine. After satisfactory reduction, a 3–5 cm long incision was made proximally at 2 cm above the apex of the greater trochanter. Under the help of the C-arm X-ray fluoroscopy machine, a guide pin was inserted into the medullary cavity through the entry point selected. The proximal end of the medullary cavity was reamed for insertion of PFNA nail. The guide pin was inserted into the femoral neck and advanced to 1 cm below the articular surface through the sleeve. When the position of the guide pin was confirmed by the C-arm X-ray fluoroscopy machine to be in the center or slightly lower part of the femoral neck in the anterior-posterior projection and in the center of the femoral neck in the lateral projection, a hole was made along the guide pin; then, a spiral blade was inserted, rotated in a clockwise manner, and locked. The distal screw was statistically tightened by bolts and nuts. Surgical site was flushed, and the incision was sutured. In the combined treatment group, in addition to the surgical procedure, a microexternal fixator was used. Precisely, after continuous epidural or general anesthesia, the affected limb was placed on the traction frame. After satisfactory reduction was achieved, surgical site was routinely disinfected, and a 3–5 cm long incision was made proximally at 2 cm above the apex of the greater trochanter. The skin, subcutaneous tissue, and tensor latissimus muscle were cut open, and coronal plane femoral intertrochanteric fracture blocks were fastened together with 3.2 mm sized threaded Steinman's pins to the femoral head to avoid the opening of the greater trochanter or the separation of anterior and posterior fracture blocks during reaming of the femoral medullary cavity. Then, routine PFNA internal fixation was performed. After incision closure, a self-designed microexternal fixator was installed on the two threaded Steinman's pins. The two threaded Steinman's pins were put close together. The fixing screws were tightened, and Steinman's pins were fastened. To implement reduction of fracture ends, distance between fracture blocks less than 2 mm, cervical trunk angle 120–140°, and varus angle less than 10° should be met.

The article "Treatment of Coronal Plane Femoral Intertrochanteric Fractures with a Microexternal Fixator Combined with Proximal Femoral Nail Antirotation" was retracted in 2023. Reasons: signs of a paper mill; suspected computer-generated content; unreliable results or conclusions; concerns about the data.

### 2.4. Postoperative Management

Patients were intravenously administered antibiotics once every 8 hours within 24 hours after surgery. At 12 hours after surgery, a calf venous pump was applied, and lower-extremity active and passive contraction training was performed to prevent deep venous thrombosis of both lower limbs. In the combined treatment group, care should also be taken to Steinman's pins and surrounding skin. The surrounding skin was scrubbed with iodophor once every 2-3 days. The site for guide pin insertion was wrapped with sterile gauze. According to the degree of fracture and fixation, Steinman's pins were removed at 4–6 weeks after surgery. Hip function exercise and partial weight-bearing gait exercise were performed starting 1-2 weeks after surgery. Weight-bearing gait exercise was performed starting 6–8 weeks after surgery. To understand fracture healing, X-ray examination of proximal femur was performed once every 15 days in the first month after surgery and once every 1 month in the subsequent 6 months.

### 2.5. Outcome Measures and Evaluation Criteria

Operative time, amount of intraoperative blood loss, postoperative length of hospital stays, fracture healing time, hip joint function (Harris hip score), activities of living ability (modified Barthel index), and postoperative complications (incision infection, hip varus, femoral head necrosis, limb shortening, and rotary knife cutting femoral head) were compared between control and combined treatment groups. At 3 months after surgery, hip function was evaluated using Harris hip score from the dimensions including pain, function (presence of limp, use of support devices, walking distance, socks and shoes, stair climbing, public transportation, and sitting), deformity of affected limbs, and motion of hip joint, with a full score of 100 points [7]. Hip function was rated excellent, good, fair, and poor with the Harris hip score ≥90 points, 80–89 points, 70–79 points, and <70 points, respectively. The excellent and good rate = (the number of patients with excellent hip function and the number of patients with good hip function)/total number of patients ×100%. At 3 months after surgery, activities of living ability were evaluated using the modified Barthel index from the dimensions including feeding, bathing, grooming, dressing, bowels, bladder, toilet use, transfers (bed to chair and back), mobility (on level surfaces), and stairs, with the full score of 100 points. A higher score indicates greater activities of living ability [8].

The article "Treatment of Coronal Plane Femoral Intertrochanteric Fractures with a Microexternal Fixator Combined with Proximal Femoral Nail Antirotation" was retracted in 2023. Reasons: signs of a paper mill; suspected computer-generated content; unreliable results or conclusions; concerns about the data.

### 2.6. Statistical Analysis

All data were statistically analyzed using SPSS 22.0 software. Count data were expressed as (*n*, %). The chi-square test was used for comparison between groups. Measurement data were expressed as the mean ± SD. The two independent samples *t*-test was used for comparison between groups.

## 3. Results

### 3.1. Comparisons of Operative Outcomes between Combined Treatment and Control Groups

Fracture healing time in the combined treatment group was significantly shorter than that in the control group (*P* < 0.05). There were no significant differences in operative time, intraoperative blood loss, and postoperative length of hospital stay between the two groups (*P* > 0.05).  Table 1 provides the comparisons of postoperative outcomes between combined treatment and control groups.

### 3.2. Comparisons of Hip Function and Activities of Daily Living between Combined Treatment and Control Groups

Before surgery, there were no significant differences in Harris hip score and MBI between combined treatment and control groups (both *P* > 0.05). At 6 months after surgery, Harris hip score and MBI in each group were significantly increased compared with before surgery (*P* < 0.05). The increases in the combined treatment group were greater than those in the control group (both *P* < 0.05).  Table 2 provides the comparisons of Harris hip score and modified Barthel index between before and after surgery.

### 3.3. Comparison of Hip Function Excellent and Good Rate between Combined Treatment and Control Groups

The hip function excellent and good rate in the combined treatment group was significantly higher than that in the control group (83.33% > 66.67%, *P* < 0.05).  Table 3 provides the comparison of hip function excellent and good rate between combined treatment and control groups.

### 3.4. Comparison of Postoperative Complications between Combined Treatment and Control Groups

After surgery, 1 case had displacement of fracture because of internal fixation failure, 1 case had hip varus, and 1 case had limb shortening in the control group. By contrast, 1 case had hip varus and no patients had internal fixation failure or limb shortening in the combined treatment group. There was no significant difference in the incidence of postoperative complications between combined treatment and control groups (5% vs. 1.67%, Χ^2^ = 1.035, *P* > 0.05). Figures 1–3 show the typical cases.

The article "Treatment of Coronal Plane Femoral Intertrochanteric Fractures with a Microexternal Fixator Combined with Proximal Femoral Nail Antirotation" was retracted in 2023. Reasons: signs of a paper mill; suspected computer-generated content; unreliable results or conclusions; concerns about the data.

## 4. Discussion

Coronal plane femoral intertrochanteric fractures are mostly caused by violence, which are a special type of femoral intertrochanteric fractures [9–11]. Internal fixation is usually used for clinical treatment of coronal plane femoral intertrochanteric fractures. PFNA is a kind of intramedullary fixation material that is characterized by good compliance, small incision, and less bleeding, which are suitable for older adults with osteoporosis [12, 13]. PFNA has been widely used to treat coronal plane femoral intertrochanteric fractures. However, because coronal plane femoral intertrochanteric fractures are extremely unstable, application of PFNA alone for treatment of such fractures can result in a high failure rate and adverse reactions such as intramedullary nail loosening and poor reduction, which affect the recovery of hip joint function [14, 15]. Therefore, it is very important to find an ideal reduction method or internal fixation instrument.

In this study, we designed a novel microexternal fixator. This fixator has advantages including ease in operation, less trauma, and reliable fixation. We used the novel microexternal fixator to manage coronal plane femoral intertrochanteric fractures, analyzed the therapeutic effects according to the special biomechanical characteristics of femoral intertrochanteric fractures and many years of clinical experience in the treatment of femoral intertrochanteric fractures, and preliminarily investigated the operative details.

Results from this study showed that there were no significant differences in operative time, intraoperative blood loss, postoperative length of hospital stay, and postoperative complications between the combined treatment and control groups. Fracture healing time in the combined treatment group was significantly shorter than that in the control group. At 6 months after surgery, Harris hip score and MBI in each group were significantly increased compared with before surgery, and the increases in the combined treatment group were significantly greater than those in the control group. At 6 months after surgery, hip function excellent and good rate in the combined treatment group were significantly greater than that in the control group (83.33% > 66.67%, *P* < 0.05). These findings suggest that compared with PFNA alone, PFNA combined with a microexternal fixator for treatment of coronal plane femoral intertrochanteric fractures can accelerate fracture healing without obviously increasing operative time, intraoperative blood loss, postoperative length of hospital stay, and the risk of postoperative complications, can promote the recovery of hip function, and improve the quality of life after surgery.

The article "Treatment of Coronal Plane Femoral Intertrochanteric Fractures with a Microexternal Fixator Combined with Proximal Femoral Nail Antirotation" was retracted in 2023. Reasons: signs of a paper mill; suspected computer-generated content; unreliable results or conclusions; concerns about the data.

PFNA is a modification of proximal femoral intramedullary nail and has the following advantages when applied to manage femoral intertrochanteric fractures: (a) the original two lag screws changed to one spiral blade, and the percussion method is adopted during the surgery. This not only reduces intraoperative bone loss but also compresses the cancellous bone in the femoral head and increases the anchoring force [16–18]. (b) The spiral blade can be locked by itself with strong holding force, which can play the role of antirotation [19]. (c) The main nail of PFNA has strong intramedullary stability. (d) Operation is often completed through a small incision. It is easy to operate and minimally invasive [20]. Coronal plane femoral intertrochanteric fractures have no obvious advantages in terms of biomechanics and operation. Biochemically, the fracture lines of femoral intertrochanteric fractures are at the coronal level, which destroys the continuity of bone cortex in the lateral wall of the femur, leading to unstable PFNA fixation [21].

The difficult point in operation is that the coronal fracture line is often passed when creating an operative incision and placing the main screw during surgery, leading to the anterior and posterior separation of the coronal fracture blocks. Some scholars used reduction forceps for temporary fixation, but the femoral trochanter is the cancellous bone, and therefore, it is easily clamped into the medullary cavity by the reduction forceps, leading to a difficulty in reaming of the proximal femur [22–24]. If the coronal plane femoral intertrochanteric fracture blocks are not fixed after successful nail fixation, shift occurs easily again after surgery, resulting in internal fixation failure, finally leading to nonunion or delayed healing of the fracture. If the internal fixation device is placed improperly, it will aggravate the separation of fracture blocks and lead to the failure of internal fixation. Tong et al. also expanded the incision in the proximal lateral femur and fixed the fracture blocks with steel plates [25]. This worsens the injury to the soft tissue around the incision and is conflicted with the concept of minimal invasion of the intramedullary system. The microexternal fixator is a tool that provides minimally invasive fracture fixation. PFNA combined with the microexternal fixator is used to treat coronal plane femoral intertrochanteric fractures. The microexternal fixator is composed of an upper gusset plate, a lower gusset plate (I), Steinman's pin, a bolt, and a nut. A space pin (I) is installed on the upper gusset plate. Multiple arc grooves (I) are created symmetrically on both sides of the upper gusset plate. A central hole is created in the center of the upper gusset plate and the center of the lower gusset plate (I). A pinhole is created in the lower gusset plate (I). Multiple arc grooves (II) are created symmetrically on both sides of the lower gusset plate (I). Steinman's pins pass across the arc grooves (I) and arc grooves (II) and are tightened by bolts and nuts, which provides overall fixation and angular stability as well as firm fixation of the fracture blocks. This conforms to the biological characteristics of the human body, resists the tensile stress of the separation of the fracture surface, and makes up for the particularity and complexity of coronal plane femoral intertrochanteric fractures. This method has characteristics including simple operation, minimal invasion, reliable fixation, and a small number of complications, contributing to fracture healing and functional recovery.

The article "Treatment of Coronal Plane Femoral Intertrochanteric Fractures with a Microexternal Fixator Combined with Proximal Femoral Nail Antirotation" was retracted in 2023. Reasons: signs of a paper mill; suspected computer-generated content; unreliable results or conclusions; concerns about the data.

This study has a few limitations: the sample size is too small, and the follow-up time is too short, which should be improved continuously by adopting long-term follow-up examinations; this study lacked a randomized control group, which should be improved; and the factors that affect the prognosis of coronal plane femoral intertrochanteric fractures are not probed into, which should investigate the factors that affect prognosis.

## 5. Conclusion

Taken together, compared with PFNA alone, a microexternal fixator combined with PFNA for the treatment of coronal plane femoral intertrochanteric coronal fractures can shorten fracture healing time and improve hip function and activities of living ability, but it cannot greatly increase operative time, the amount of intraoperative blood loss, or the risk of postoperative complications.

## Figures and Tables

**Figure 1:** Surgical approach for left femoral intertrochanteric fracture.

**Figure 2:** Surgical nail placement process.

**Figure 3:** Preoperative and postoperative X-ray comparison.

**Table 1:** Comparisons of postoperative outcomes between combined treatment and control groups ($\bar{x}$ ± *s*).

Group	*n*	Operative time (min)	Intraoperative blood loss (mL)	Postoperative length of hospital stay (d)	Fracture healing time (week)
Control	60	58.13 ± 12.35	150.24 ± 28.75	8.35 ± 1.78	20.89 ± 2.33
Combined treatment	60	62.72 ± 13.74	155.36 ± 35.74	9.04 ± 2.37	17.12 ± 2.16
*t*		1.924	0.865	1.803	9.191
*P*		*P* > 0.05	*P* > 0.05	*P* > 0.05	*P* < 0.05

The article "Treatment of Coronal Plane Femoral Intertrochanteric Fractures with a Microexternal Fixator Combined with Proximal Femoral Nail Antirotation" was retracted in 2023. Reasons: signs of a paper mill; suspected computer-generated content; unreliable results or conclusions; concerns about the data.

**Table 2:** Comparisons of Harris hip score and modified Barthel index between before and after surgery ($\bar{x}$ ± *s*).

Group	Harris hip score (point)		Modified Barthel index (point)	
	Before surgery	6 months after surgery	Before surgery	6 months after surgery
Control	51.85 ± 7.33	81.94 ± 8.22^#^	31.27 ± 4.19	79.52 ± 7.91^#^
Combination	50.91 ± 8.14	87.76 ± 9.83^#^	32.36 ± 4.28	84.35 ± 8.12^#^
*t*	0.665	3.518	1.410	3.300
*P*	*P* > 0.05	*P* < 0.05	*P* > 0.05	*P* < 0.05

^#^ *P* < 0.05 vs. before surgery in the same group.

**Table 3:** Comparison of hip function excellent and good rate between combined treatment and control groups (*n* (%)).

Group	Excellent	Good	Fair	Poor	Total effective rate
Control	16 (26.67)	24 (40.00)	16 (26.67)	4 (6.67)	40 (66.67)
Combined treatment	27 (45.00)	23 (38.33)	10 (16.67)	0 (0)	50 (83.33)
Χ^2^					4.444
*P*					<0.05

## Data Availability

The simulation experiment data used to support the findings of this study are available from the corresponding author upon request.
